This article has been retracted.

# MiRNA‐545 negatively regulates the oncogenic activity of EMS1 in gastric cancer

**DOI:** 10.1002/cam4.1520

**Published:** 2018-05-07

**Authors:** Min Ma, Juanxia Zhao, Qunfeng Wu, Ke Xiao, Shuang Li, Haizhen Zhu, Chen Liu, Hailong Xie, Chaohui Zuo

**Affiliations:** ^1^ The Affiliated Cancer Hospital of Xiangya School of Medicine Central South University Hunan Cancer Hospital Changsha Hunan 410013 China; ^2^ Institute of Cancer Research School of Medicine University of South China Hengyang Hunan 421001 China; ^3^ Department of Pathology and Laboratory Medicine New Jersey Medical School Rutgers, The State University of New Jersey Newark New Jersey 07103; ^4^ Department of Molecular Medicine College of Biology State Key Laboratory of Chemo/Biosensing and Chemometrics Hunan University Changsha Hunan 410082 China

**Keywords:** Cell proliferation, EMS1, EMT process, gastric cancer, miR‐545

## Abstract

Gastric cancer (GC) is a common malignant tumor of the digestive system. In addition, GC metastasis is an extremely complicated process. In this article, high expression levels of EMS1 mRNA and protein were found to be positively correlated with an enhanced malignant potential of GC cells and a poor clinical prognosis of GC patients. Interestingly, the expression levels of EMS1 mRNA and protein in GC cells were inhibited by microRNA‐545 (miR‐545), which was identified by a bioinformatics analysis. The expression level of miR‐545 in carcinoma tissues was significantly lower than that in para‐carcinoma tissues. The proliferation and epithelial‐mesenchymal transition (EMT) of GC cells were suppressed by exogenous oligonucleotides of miR‐545 mimics. In addition, the expression levels of EMT‐associated markers were altered with the expression of miR‐545. Notably, the growth rates of tumors in nude mice were seriously restrained by an intratumoral injection of oligonucleotides of the miR‐545 mimics. These results suggest a negative regulatory role of miR‐545 on the oncogenic activity of EMS1. In addition, EMS1 and miR‐545 may be potential biomarkers for GC diagnosis. Synthesized oligonucleotides of miR‐545 mimics may be developed as important gene medicines for GC therapy in the future.

## Introduction

Gastric cancer (GC) is a common malignant carcinoma of the digestive system. According to a 2015 report, 679,100 patients were diagnosed with newly found GC in China, accounting for 15.8% of the newly confirmed cancer patients 1. In addition, 498,000 of these cases resulted in death, accounting for 17.7% of all deaths from malignant neoplasms. Fortunately, the death rate of GC has declined in recent years due to the improved environment and dietary habits and early diagnosis in the clinic 2. However, comprehensive diagnosis of GC at an early stage is difficult due to limited availability of medical care 3. In addition, effective therapy for the frequent metastasis of GC to lymph nodes and distant sites is lacking.

GC metastasis is an extremely complicated biological process. The abnormal expression of oncogenes is considered a precondition for the occurrence of GC metastasis. A high frequency of DNA amplification at the chromosome 11q13 region in the genome usually leads to activation of oncogenes 4, 5, 6. EMS1 and cyclin D1 were discovered at chromosome 11q13 in human breast and head and neck cancer cells 7, 8, 9. Cortactin, a protein encoded by EMS1, strongly binds with F‐actin in the cortical region of cells 10, 11. Cortactin plays significant roles in cell mobility, cytoskeleton remodeling, and cancer metastasis and is highly expressed in neoplasms, including esophageal squamous cancer 12, squamous cell carcinoma of the head and neck 13, colorectal cancer 14, pancreatic cancer 15, renal cell carcinoma 16, and melanoma 17. Reinforcement of cell motility is an important mechanism of tumor invasion 18. Therefore, cortactin plays an important role in cancer invasion and metastasis.

As a cluster of endogenous single‐stranded and small molecule RNAs that are 18~25 nucleotides in length, microRNAs (miRNAs) provide new hope for cancer therapy 19. The regulatory activity of miRNAs is nearly 10‐fold that of synthetic siRNAs without associated changes in the sequences of target genes; this indicates the advantages of miRNAs in gene therapy 20, 21. Notably, increasing achievements have been made in revealing the correlation between miRNAs and neoplasms. Differential expression of miRNAs has been repeatedly discovered between carcinoma and para‐carcinoma tissues, suggesting the relevance of miRNAs in tumorigenesis 22, 23, 24.

MiRNAs can localize to the cell nucleus to regulate the expression of crucial genes correlated with carcinomas that influence cancer cell proliferation, apoptosis, migration, metastasis, invasion, adhesion to matrix, and angiogenesis. However, no miRNAs have been reported to act on the oncogene EMS1. In this article, EMS1 expression was found to be positively correlated with a poor clinical prognosis of GC. Through a bioinformatics analysis, miR‐545 was found to effectively inhibit EMS1 expression and cell proliferation, epithelial‐mesenchymal transition (EMT), and tumor growth in GC. EMS1 and miR‐545 may be potential biomarkers for GC diagnosis. In addition, miR‐545 may be a significant target for GC therapy.

## Materials and Methods

### Cell culture

Human normal gastric mucosal cells GES‐1 and GC cells BGC‐823, MGC‐803, HGC‐027, and SGC‐7901 were purchased from BOSTER (Wuhan, Hubei, China) or the Cell Bank of the Chinese Academy of Sciences (Shanghai, China). Cells were cultured in DMEM (Thermo Fisher Scientific, Waltham, MA) supplemented with 10% (v/v) FBS, penicillin, and streptomycin (Thermo Fisher Scientific).

### Transfection of miRNAs

The oligonucleotides of miR‐545 mimics, inhibitors, and negative controls (NC) are summarized in Table 1; these were synthesized at Sangon Biotech (Shanghai, China). GC cells were seeded in a six‐well plate (Corning Incorporated, Corning, NY) at 50–60% confluence. After cultivation for 24 h, the cells were transfected with 100 nmol/L miRNAs using Lipofectamine^™^ 2000 (Thermo Fisher Scientific). The transfection efficiency and expression levels of miR‐545 and EMS1 were evaluated by quantitative real‐time polymerase chain reaction (qRT‐PCR) or Western blotting.

**Table 1:** Sequences of miR‐545 oligonucleotides

Oligonucleotides	Sequences (5′ to 3′)
miR‐545 mimics	UCAGCAAACAUUUAUUGUGUGC
miR‐545 inhibitor	GCACACAATAAATGTTTGCTGA
NC group	UUCUCCGAACGUGUCACGUdTdT

### PCR experiments

From January 2016 to April 2016, 20 pairs of GC tissues were collected at Hunan Cancer Hospital. All procedures performed in the study involving human participants were approved by the Institutional Review Board of Hunan Cancer Hospital affiliated with Xiangya Medical School (Changsha, China) in accordance with the Declaration of Helsinki. All human tissue samples were obtained with informed consent and approval from the Ethics Committee of Hunan Cancer Hospital and the Affiliated Cancer Hospital of Xiangya Medical School.

The total RNA of the GC cells and tissues was extracted using TRIzol reagent (Thermo Fisher Scientific). Reverse transcription PCR (RT‐PCR) and qRT‐PCR of the mRNA was performed using the PrimeScript^™^ RT reagent Kit with gDNA Eraser (Takara, Tokyo, Japan) and the SYBR^®^ Premix Ex Taq^™^ II (Tli RNaseH Plus) (Takara). To determine miR‐545 expression, the total RNA was treated with the RNase‐free DNase (Promega, Madison, WI). RT‐PCR and qRT‐PCR were conducted using the All‐in‐One^™^ miRNA qRT‐PCR Detection System (GeneCopoeia, Rockville, MD). The specific primer of miR‐545 was TCA GCA AAC ATT TAT TGT GTGC. The primer of the internal control U6 was purchased from GeneCopoeia. The relative expression level was normalized to the NC group. The specific primers (forward primer: CGC CGT TGG CTT TGA GTA TC; reverse primer: CTG CCT CTC CGA CTG AAC AC) for EMS1 were used for qRT‐PCR. The internal control was *β*‐actin (forward primer: TCC CTG GAG AAG AGC TAC GA; reverse primer: AGC ACT GTG TTG GCG TAC AG).

### Western blotting

The cell and tissue lysates were obtained using the RIPA buffer and quantified by the BCA method. The proteins were run on an SDS‐PAGE gel and transferred onto a PVDF membrane. The following antibodies were used: rabbit anti‐EMS1 (CST, Danvers, MA), mouse anti‐*β*‐actin (Sigma, Darmstadt, Germany), EMT Antibody Sampler Kit (CST), goat anti‐mouse (Merck Millipore, Darmstadt, Germany), and goat anti‐rabbit (CST). The protein bands were detected using SuperSignal^™^ West Pico Chemiluminescent Substrate (Thermo Fisher Scientific).

### Immunochemistry

A total of 48 GC tissues were used for immunochemistry staining. Tissues were routinely embedded in paraffin, cut into slices and dewaxed. The slices were then routinely hydrated step by step with decreasing concentrations of alcohol solution. After blocking with 3% H_2_O_2_, antigens of the slices were repaired in 0.01 mol/L citrate buffer at 95°C for 15 min. Then, the slices were blocked with normal goat serum at room temperature for 20 min and sequentially incubated with antibodies at room temperature for 1 h. DAB was used as a chromogenic reagent. Images of the stained slices were captured using inverted optical microscopy.

### MTT assay

Overall, 1 × 10^4^ transfected GC cells in 100 *μ*L of culture medium were seeded per well in a 96‐well plate. After cultivation, 10 *μ*L of 5 mg/mL MTT solution was added to the culture medium and incubated for 4 h. Then, the culture medium was carefully removed and replaced with 150 *μ*L of DMSO. The OD value at 490 nm was measured for analysis. All experiments were repeated three times.

### Wound healing assay

The transfected cells were seeded in a six‐well plate at 50–60% confluence and cultivated for 24 h. After host starvation for another 24 h, the cells were scratched using a standard 10‐*μ*L pipette tip and cultivated in DMEM without FBS. Images of the wound healing process were captured for analysis.

### Transwell assay

The 24‐well chambers with 8.0‐*μ*m PET membrane pores (Corning Incorporated) were used to evaluate the migration ability of GC cells. After transfection for 24 h, the cells were starved with serum‐free DMEM for another 24 h. Then, 650 *μ*L of DMEM supplemented with 10% (v/v) FBS was added to the lower chamber of the Transwell, and 100 *μ*L of serum‐free DMEM with 1 × 10^5^ transfected cells was added to the upper chamber. After cultivation for 24 h, the transmigrated cells were fixed with methyl alcohol and stained with 0.2% (m/v) crystal violet. Images of the transmigrated cells were captured for analysis.

### Adhesion assay

A 96‐well plate was coated with 30 *μ*L of 40 *μ*g/mL collagen I for 12 h, rinsed with PBS, and dried at room temperature. After transfection for 24 h, the cells were starved with serum‐free DMEM for 8 h. To conduct adhesion assays, the cells were detached using 10 mmol/L EDTA for 10 min, washed with DMEM, and resuspended at a density of 2 × 10^5^ cells/mL in DMEM with 0.1% (m/v) BSA. Overall, 100 *μ*L of cell suspension was added to the coated wells and cultivated at 37°C for 20 min. The nonadherent cells were washed off using serum‐free DMEM. The adherent cells were cultured in DMEM supplemented with 10% (v/v) FBS at 37°C for 4 h and examined by MTT.

### Tumor xenograft and intratumoral injection

The animal experiments performed in this study were approved by the Animal Care and Experiment Committee of Hunan Cancer Hospital. Every effort was made to minimize the pain of the mice. A total of 18 four‐week‐old female athymic BALB/C nude mice (SJA, Hunan, China) were fed under standard conditions at the animal care facility. Overall, 1 × 10^7^ BGC‐823 cells in 200 *μ*L of sterile PBS were administered to the BALB/c nude mice by subcutaneous injection.

After tumor formation for 2 weeks, the mice were separated into three groups (*n* = 6 each). Exogenous oligonucleotides of miR‐545 were administered to the mice every 3 days through intratumoral injection according to the methods described in previous reports 25, 26, 27. In brief, 100 *μ*L of 85 nmol/L siRNA in PBS was injected into the subcutaneous tumors every 3 days. Mice were sacrificed 3 weeks later. The tumor volume was calculated according to the following formula: tumor volume (mm^3^) = 0.5 × length × width^2^.

### Ethical standards

The execution of the animal experiments was approved by the Animal Care and Experiment Committee of Hunan Cancer Hospital. Human tissues were obtained with informed consent and approval from the Ethics Committee of Hunan Cancer Hospital.

### Statistical analysis

Student's *t*‐test and one‐way analysis of variance were used for statistical analysis. GraphPad Prism 5.0 (GraphPad Software, La Jolla, CA) was used to draw graphs. The results are expressed as the mean ± standard deviation (SD). A statistically significant difference was defined as follows: *P <* *0.05, **P <* *0.01, and ***P <* *0.001.

## Results

### High expression of EMS1 is tightly associated with a poor prognosis of GC

To uncover the clinical significance of EMS1 in GC, the expression profile of EMS1 was examined by qRT‐PCR and Western blotting. The expression level of EMS1 mRNA in the GC cells BGC‐823, MGC‐803, SGC‐7901, and HGC‐027 was significantly higher than that of normal GES‐1 gastric mucosal cells (Fig. 1A). Similarly, the protein level of EMS1 in GC cells was much more abundant than that in GES‐1 cells (Fig. 1B). Notably, EMS1 mRNA and protein expression were highly associated with the degree of malignancy, suggesting upregulated expression of EMS1 in GC cells.

**Figure 1:** Expression profile of EMS1 in GC. (A and B) The expression profile of EMS1 in GC cells, as assayed by qRT‐PCR and Western blotting. (C) Scatter diagram showing the differential expression level of EMS1 in carcinoma tissues (CTs) and para‐carcinoma tissues (para‐CTs), as assayed by qRT‐PCR. (D) The expression level of EMS1 in CTs and para‐CTs, as assayed by Western blotting. (E) The expression level of EMS1 was evaluated according to the following four degrees based on immunochemistry: score 0: no stained cells or stained cells in the nucleus; score +: stained cells ≤25%; score ++: stained cells >25% and ≤50%; and score +++: stained cells >50%. Representative pictographs are depicted at ×400.

We then extended our findings in cell lines to clinical samples by analyzing the expression levels of EMS1 mRNA and protein in 20 pairs of human para‐carcinoma and carcinoma GC tissues. The para‐carcinoma tissues were the gastric tissues with 2 cm away from the edge of carcinoma tissues. Compared with the para‐carcinoma tissues, over 50% of the GC tissues highly expressed EMS1 mRNA (Fig. 1C), and EMS1 protein in the carcinoma tissues was more abundant (Fig. 1D). To further confirm our discovery, EMS1 protein in 48 GC tissue samples was detected by immunochemistry and evaluated as four degrees (Fig. 1E). It was obvious that EMS1 protein mainly existed in the cytoplasm. EMS1 protein was highly expressed in poorly differentiated GC tissues and was lowly expressed in moderately differentiated GC tissues. In contrast, almost no expression of the EMS1 protein was observed in well‐differentiated GC tissues and para‐carcinoma tissues. These results demonstrated the oncogenic role of EMS1. Owing to the shortage of late‐stage GC cases, no difference was found in the undifferentiated GC tissues. By analyzing the clinical pathological findings of GC patients, the expression level of EMS1 was shown to be highly correlated with lymphatic metastasis and TNM stage (Table 2). Therefore, high EMS1 expression may result in metastasis and a poor prognosis in GC. The univariate analyses of overall survival confirmed the correlation between EMS1 expression and T stage, lymphatic metastasis, distant metastases, and TNM stage (Table 3). Because of the limited samples, the multivariate analyses of overall survival only showed a close relationship between EMS1 expression level and TNM stage. In conclusion, high EMS1 expression promotes the deterioration of GC and predicts the occurrence of lymphatic metastasis and distant metastases, which results in a poor prognosis.

**Table 2:** Clinicopathologic features among different expression groups of EMS1

Parameters	0	+	++	+++	*M*
	*N*	*N*	*N*	*N*	
Sex					
Male	2	4	11	17	0.266
Female	1	4	6	3	
Age					
<60	2	6	12	12	0.857
≥60	1	2	5	8	
Lauren type					
Intestinal type	2	3	6	8	0.666
Diffuse type	1	5	8	11	
Mixed type	0	0	3	1	
Tumor size					
<4.3 cm	3	7	10	10	0.147
≥4.3 cm	0	1	7	10	
Tumor location					
Gastric fundus and cardiac	1	1	4	6	0.640
Gastric body	0	0	3	4	
Gastric antrum	2	7	10	10	
Histological grade					
Well‐differentiated	1	0	1	3	0.430
Moderately differentiated	1	3	5	3	
Poorly differentiated	1	5	9	14	
Undifferentiated	0	0	2	0	
T staging					
T1	0	3	1	1	0.001
T2	3	3	3	1	
T3	0	2	13	15	
T4	0	0	0	3	
Presence of LN metastasis					
No	2	6	5	2	0.004
Yes	1	2	12	18	
Presence of distant metastases					
No	3	8	17	18	0.432
Yes	0	0	0	2	
Borrmann type					
I	0	0	1	0	0.472
II	1	4	13	9	
III	2	4	3	10	
IV	0	0	0	1	
Presence of vascular and nerve bundle					
No	2	5	6	7	0.415
Yes	1	3	11	13	
TNM stage					
I	2	4	3	0	0.013
II	1	3	3	4	
III	0	1	11	14	
IV	0	0	0	2	

**Table 3:** Univariate and multivariate analyses of overall survival in GC patients

	Univariate analyses			Multivariate analyses		
	HR	95% CI	*P*	HR	95% CI	*P*
T staging	3.435	1.203–9.810	0.021			
Presence of LN metastasis	5.995	1.393–25.804	0.016			
Presence of distant metastasis	7.639	1.535–38.019	0.013			
The expression level of EMS1	3.418	1.570–7.440	0.002	2.509	1.087–5.790	0.031
TNM staging	4.256	1.7896–10.145	0.001	3.188	1.318–7.771	0.010

### MiR‐545 negatively regulates EMS1 expression in GC

Considering the long 3′ UTR region of EMS1, we speculated that the expression of EMS1 might also be regulated by miRNAs. Through a bioinformatics analysis on the website miRwalk (http://zmf.umm.uni-heidelberg.de/apps/zmf/mirwalk2/index.html) 28, 29, miRNAs, including miR‐182, miR‐501‐3p, miR‐502‐3p, miR‐545, miR‐329, miR‐603, miR‐326, were predicted to regulate EMS1 expression. In addition, miR‐545 had the highest grade and was chosen for our research. In contrast to EMS1 expression, miR‐545 was highly expressed in GES‐1 cells, whereas it was lowly expressed in GC cells (Fig. 2A). In addition, the expression level of miR‐545 in 80% of GC tissues was significantly lower than that in para‐carcinoma tissues (Fig. 2B). These results suggested a tumor suppressor role of miR‐545 in GC.

**Figure 2:** The expression of EMS1 in GC cells was controlled by miR‐545. (A) Expression profile of miR‐545 in GC cells, as assayed by qRT‐PCR. (B) Scatter diagram showing the differential expression of miR‐545 in CTs and para‐CTs, as assayed by qRT‐PCR. (C~E) Histograms showing the expression level of miR‐545 and EMS1 in BGC‐823 and SGC‐7901 cells after transfection with miR‐545 oligonucleotides, as assayed by qRT‐PCR and Western blotting. (F) Proliferation of GC cells after transfection with miR‐545 oligonucleotides, as assayed by MTT.

To evaluate the regulatory role of miR‐545 in EMS1 expression, the synthesized oligonucleotides of miR‐545 were transiently transfected into the cancer cell lines BGC‐823 and SGC‐7901. Compared with that of the NC group, the expression level of miR‐545 in inhibitor group was significantly reduced to less than 10%, while it was upregulated over 240‐ and 200‐fold in the mimics group (Fig. 2C). In contrast, the expression level of EMS1 mRNA was upregulated in the inhibitor group, while it was downregulated in the mimics group (Fig. 2D). In addition, the protein expression of EMS1 in GC cells was much more abundant in the miR‐545 inhibitor group but was lower in the miR‐545 mimics group than in the NC group (Fig. 2E). Therefore, EMS1 expression in GC cells can be effectively inhibited by upregulating miR‐545. Cell proliferation was significantly enhanced in the miR‐545 inhibitor group, while it was markedly suppressed in the miR‐545 mimics group (Fig. 2F). In conclusion, miR‐545 inhibits EMS1 expression and GC cell proliferation, suggesting a suppressive role of miR‐545 on the oncogenic activity of EMS1.

### MiR‐545 suppresses EMT in GC cells

Considering the acceleratory effect of EMS1 in cancer metastasis, we examined the influence of miR‐545 on EMT. The wound healing speed of GC cells was accelerated in the miR‐545 inhibitor group, while it was decreased in the miR‐545 mimics group (Fig. 3A and B). These results were further confirmed by Transwell assays. The number of migrating GC cells was increased in the miR‐545 inhibitor group, while it was reduced in the miR‐545 mimics group (Fig. 3C and D). The ability of GC cells to adhere to the matrix, as examined by adhesion assays, was enhanced in the miR‐545 inhibitor group, while this ability was diminished by oligonucleotides of miR‐545 mimics (Fig. 3E). Therefore, miR‐545 restrains the migration and adhesion abilities of GC cells.

**Figure 3:** EMT in GC cell lines BGC‐823 and SGC‐7901 was regulated by miR‐545. (A and B) Alteration of migratory behavior of GC cells after transfection with miR‐545 oligonucleotides, as assayed by wound healing. (C and D) Migration ability of GC cells after transfection with miR‐545 oligonucleotides, as evaluated by Transwell assays. (E) Ability of GC cells to adhere to the matrix, as examined by adhesion assays. (F) The expression levels of EMT‐associated markers, as assayed by Western blotting.

To explain the abovementioned biological phenomena, EMT‐associated markers were examined by Western blotting. After transfection with oligonucleotides of miR‐545 inhibitors, the epithelial marker E‐cadherin was downregulated, while the mesenchymal markers vimentin, *β*‐catenin, and slug were upregulated (Fig. 3F), resulting in an enhanced migration ability of GC cells. However, the protein expression of these markers was reversed after transfection with oligonucleotides of miR‐545 mimics. In conclusion, miR‐545 not only inhibits cell proliferation but also suppresses EMT in GC cells, which may result from the effects of miR‐545 controlling EMS1 expression.

### Exogenous oligonucleotides of miR‐545 mimics efficiently inhibit tumor growth in vivo

To evaluate the therapeutic potential of miR‐545 in vivo, BGC‐823 GC cells were injected subcutaneously into female BALB/C nude mice. Exogenous oligonucleotides of miR‐545 were also administered to the mice through intratumoral injection. Compared with the tumors in the NC group, the observed tumors were smaller in the miR‐545 mimics group but were larger in the miR‐545 inhibitor group (Fig. 4A). Statistical analysis of tumor volume and weight further confirmed our observation that tumor growth was significantly inhibited by miR‐545 (Fig. 4B and C). Therefore, the growth rate of formed tumors can be suppressed by the administration of exogenous oligonucleotides of miR‐545 mimics, which confirms the therapeutic potential of oligonucleotides of miR‐545 mimics and validates the vital role of miR‐545 in controlling GC development.

**Figure 4:** MiR‐545 controlled the growth rate of formed tumors in vivo through intratumoral injection. (A) Image showing the tumors formed by BGC‐823 GC cells in mice after intratumoral injection of miR‐545 oligonucleotides. The minimum scale of the stainless steel ruler is 1 mm. (B and C) Histograms showing the statistical analysis of tumor volume and weight in (A).

## Discussion

EMT was first discovered in embryonic cells 30. In cancer, EMT is defined as the process by which cancer cells gradually downregulate the expression of cadherin‐related proteins and abnormally upregulate the expression of mesenchymal proteins 31. In addition, the cytoskeleton is altered and loses cell polarity to allow cell motility. As a result, these evolutionary mesenchymal cells are transported to and seeded in other organs via the bloodstream to develop new cancer foci. EMT is the central event in the formation of metastatic carcinomas, and transformation of the tumor microenvironment is a critical factor in facilitating EMT. TGF‐*β* plays a dominant role in altering the tumor microenvironment 32. Notably, EMS1 plays a role in TGF‐*β*‐induced EMT 33. In this study, high expression of EMS1 was found in GC tissues and was associated with the TNM stage, suggesting an association with metastatic potential and poor prognosis in GC. High EMS1 expression may be an important factor for GC diagnosis.

Worldwide, miRNAs are considered to be involved in gene regulation 34. For example, a functional variant at chromosome 3q28 promotes cell proliferation and migration by altering the binding site of miR‐140‐5p in bladder cancer 35. In addition, miR‐34a inhibits prostate cancer stem cells and metastasis by repressing CD44 expression 36, 37. Interestingly, miR‐545 was predicted to be the most efficient miRNA for regulating EMS1 expression based on a bioinformatics analysis. MiR‐545 inhibits EGFR expression and pancreatic ductal adenocarcinoma growth by targeting RIG‐I 38, 39 and enhances radiosensitivity by suppressing Ku70 expression in a Lewis lung carcinoma xenograft model 40. In this study, EMS1 expression in GC cells was found to be inhibited by oligonucleotides of miR‐545 mimics and enhanced by oligonucleotides of miR‐545 inhibitors. Therefore, miR‐545 negatively regulates EMS1 expression and GC progression. In addition, oligonucleotides of miR‐545 mimics may be developed as efficient gene medicines for GC therapy.

Owing to the accelerating function of EMS1 in cancer metastasis, miR‐545 might suppress EMT. The ability of BGC‐823 and SGC‐7901 cells to migrate and adhere to the matrix was markedly suppressed after transfection with oligonucleotides of miR‐545 mimics and was reversed by oligonucleotides of miR‐545 inhibitors, thus confirming our hypothesis. In addition, the tumor growth rate was attenuated by administering oligonucleotides of miR‐545 mimics through intratumoral injection, suggesting the therapeutic potential of miR‐545 in neoplasms. In conclusion, high expression of miR‐545 inhibits EMT in GC and the oncogenic actions of EMS1.

The importance and innovations of this study are mainly embodied by the following aspects. First, the upregulated expression of EMS1 in GC cells and tissues further confirmed the oncogenic role of EMS1, suggesting the function of EMS1 in carcinogenesis. Second, in the bioinformatics analysis, miR‐545 was found to be the first miRNA to inhibit EMS1 expression. Finally, the inhibitory effect of miR‐545 on the growth of tumors in vivo suggested the therapeutic potential of oligonucleotides of miR‐545 mimics. However, the detailed regulatory mechanisms of miR‐545 on EMS1 expression should be further explored in future research.

## Conflict of Interest

None declared.
